The article "TM4SF1 is a potential target for anti-invasion and metastasis in ovarian cancer" was published in 2019. Journal: BMC Cancer.

# TM4SF1 is a potential target for anti-invasion and metastasis in ovarian cancer

**DOI:** 10.1186/s12885-019-5417-7

**Published:** 2019-03-15

**Authors:** Caiyun Gao, Hongyu Yao, Huimin Liu, Yanying Feng, Zhijun Yang

**Affiliations:** 1 Department of Gynecologic Oncology, Affiliated Tumor Hospital of Guangxi Medical University, No.71 Hedi Road, Nanning, 530021 China; 2 Key laboratory of High-Incidence-Tumor Prevention &Treatment (Guangxi Medical University), Ministry of Education, No.22 Shuanyong Road, Nanning, 530021 China; 3 Departments of Electrocardiogram, Affiliated Tumor Hospital of Guangxi Medical University, No.71 Hedi Road, Nanning, 530021 China

**Keywords:** TM4SF1, Ovarian cancer, Invasion, Metastasis, Target

## Abstract

**Background:**

Patients with ovarian cancer commonly have a poor prognosis, owing to its invasiveness and distant metastasis. Studies have found TM4SF1 participates in regulating tumor cell invasion and migration. Therefore, it is expected to become a target for anti-invasion and metastasis in ovarian cancer.

**Methods:**

The expression of TM4SF1 in normal ovarian epithelial tissues, benign ovarian tumor tissues, primary foci of epithelial ovarian cancer and the matched lymph mode metastatic foci was detected using immunohistochemistry to analyze its association with prognosis. The expression of TM4SF1 in HO8910PM**,** SKOV3 was inhibited using RNAi, and the growth, proliferation, migration, invasion abilities of HO8910PM and SKOV3 cells and the growth of xenograft tumors in nude mice were examined.

**Results:**

(1) The positive expression rate of TM4SF1 protein in epithelial ovarian cancer tissues (90.90%) was higher than that in benign ovarian tumor tissues (65.22%) and normal ovarian epithelial tissues (31.25%), and both differences were significant (*P* < 0.05). The expression of TM4SF1 protein was positive in all metastatic lymph node foci and matched primary foci (100%). (2) The level of TM4SF1 protein expression was positively correlated with the International Federation of Gynecology and Obstetrics (FIGO) stage and histological grade. However, The positive TM4SF1 protein expression was not an independent factor of prognosis (*P* > 0.05). (3) Silencing TM4SF1 expression did not affect growth, proliferation, or cell cycle distribution but inhibited the migration and invasion abilities of HO8910PM and SKOV3 cells. Silencing TM4SF1 expression inhibited the growth of xenograft tumors in nude mice.

**Conclusion:**

TM4SF1 is a potential target for anti-invasion and metastasis in ovarian cancer.

## Background

Among malignant tumors of the female reproductive tract, ovarian cancer is the third most prevalent, and its mortality ranks fifth among female malignant tumors and first among malignant tumors of the female reproductive tract. Because early-stage ovarian cancer lacks typical clinical symptoms, approximately 2/3 of patients already have advanced stage cancer upon clinical diagnosis. Among these patients, approximately 2/3 die of tumor recurrence and metastasis within 5 years. Therefore, although the overall 5-year survival rate of ovarian cancer patients receiving standard surgery and adjuvant chemotherapy is approximately 30%, controlling tumor recurrence and distant metastasis is the key to increasing treatment efficacy and improving prognosis.

Our study group previously applied the strategy of a combination of improved serological analysis of recombinant cDNA expression libraries (SEREX) technology and suppression subtractive hybridization (SSH) technology to screen and obtain the ovarian cancer associated antigen, transmembrane 4 superfamily 1 (TM4SF1), from a cDNA library constructed from ascites cancer cells of ovarian cancer patients [1]; in addition, the autoantibody of TM4SF1 could be used for early diagnosis of ovarian cancer [2]. Several studies have already confirmed that high TM4SF1 expression in various epithelial malignant tumors can regulate cancer cell invasion and metastasis and is associated with poor prognosis [3–6]. Therefore, TM4SF1 is a potential anti-tumor therapy target. Many researchers have implemented targeted antibody therapy [7, 8], antibody-directed enzyme prodrug therapy [9], radioimmunotherapy [10], and targeted therapy with conjugated anti-tumor drugs [11] directly targeting TM4SF1.

The value of TM4SF1 as a target for anti-tumor therapy was investigated in this study by examining the expression of TM4SF1 in ovarian cancer tissues and its effects on the biological behaviors of the highly metastatic ovarian cancer cell line HO8910PM and SKOV3 cells and on the growth of xenograft tumors in nude mice.

## Methods

### Clinical data and cell culture

Fifty-five cases of patients with primary epithelial ovarian cancer (EOC), 30 cases pair-matched lymph node metastasis specimens. 23 cases of benign ovarian tumor tissues, 11 cases of normal ovarian epithelial tissues. The protocols used in our study were approved by the Ethics Committee of Affiliated Tumor Hospital of Guangxi Medical University. The EOC specimens were classified according to the FIGO stage (2014), and the clinicopathological characteristics of patients with EOC, benign ovarian tumor tissues, normal ovarian epithelial tissues are presented in Table 1. Human ovarian cancer cell lines (SKOV3, A2780, HO8910, and H08910PM) and human kidney epithelial 293 T cells were bought from cell bank of Chinese Academy of Sciences stored at Key laboratory of High-Incidence-Tumor Prevention &Treatment (Guangxi Medical University), Ministry of Education. The cells were cultured in a humidified incubator with 5% CO2 at 37 °C in RPMI1640 medium containing 10% or 20% fetal bovine serum (FBS). 5-w-old female nude mice with a body weight of 17–20 g were purchased from and fed in the experimental animal center of Guangxi Medical University.

**Table 1:** Clinicopathological characteristics of ovarian tissues

	EOC	BOT	NOT
Total cases(n)	55	23	11
FIGO		–	–
I~II	21	–	–
III~IV	34	–	–
Histological grade		–	–
Grade 1	16	–	–
Grade 2–3	39	–	–
Histological type		–	–
Serous	29	13	–
Mucinous	16	10	–
Endometrioid	8	–	–
Clear cell	2	–	–
Ascites		–	–
<500 ml	37	–	–
≥ 500 ml	18	–	–
Age(y)	21~74	23~59	28~66

*BOT* benign ovarian tumor tissues, *NOT* normal ovarian epithelial tissues

### Primers and short hairpin RNA (shRNA)

Primers were designed using the Primer 5 primer design software according to the coding sequence (CDS) of human TM4SF1 (NM_014220) in GenBank. Primers sequences are presented in Table 2.

**Table 2:** Primers sequences

	Sense	Antisense	Product
TM4SF1	5′-TTCCATTCCACAATGTGCTT-3’	5′-GGCCAGTGGAACTACACCTT-3’	101 bp
β-actin	5′- ACCGAGCGCGGCTACAGC-3’	5′- CTCATTGCCAATGGTGAT − 3’	180 bp
GAPDH	5′-GTCAAGGCTGAGAACGGGAA-3′	5′-AAATGAGCCCCAGCCTTCTC-3’	158 bp

The lentiviral plasmid containing human TM4SF1 shRNA (including the GFP reporter gene) was constructed and confirmed by Shanghai KeyGEN (China). Sequences of siRNA of TM4SF1 are presented in Table 3.

**Table 3:** siRNA of TM4SF1

NO.	Sequence
733	5′-3′: GGC UCU UGG UGG AAU UGA ATT
	UUC AAU UCC ACC AAG AGC CTT
497	5′-3′: GCG AUG CUU UCU UCU GUA UTT
	AUA CAG AAG AAA GCA UCG CTT
813	5′-3′: GCU CUC ACC AAC AGC AAU ATT
	UAU UGC UGU UGG UGA GAG CTT
NC	5′-3′: UUC UCC GAA CGU GUC ACG UTT
	ACG UGA CAC GUU CGG AGA ATT
GA	5′-3′: GUA UGA CAA CAG CCU CAA GTT
	CUU GAG GCU GUU GUC AUA CTT
Positive sequence	5′-3′:GCGATGCTTTCTTCTGTAT
Control sequence	5′-3′:TTCTCCGAACGTGTCACGT

## Methods

### Detection of TM4SF1 expression using immunohistochemistry (SP method)

Pre-selected paraffin sections were deparaffinized and dehydrated. Antigen retrieval was performed using the high-pressure method in 0.01 mol/L citrate buffer for 20 min. Sections were blocked in goat serum for 15 min and incubated with 1:2000 rabbit anti-human TM4SF1 (Abcam, USA) at 4 °C overnight. Sections were then incubated with goat anti-rabbit secondary antibody (CST, USA) at 37 °C for 1 h and developed using DAB (Beijing ZSGB-BIO, China) for 1 min. Sections were air- dried and mounted. Breast cancer tissues were used as the positive control, and as the negative control, the primary antibody was replaced with PBS.

The presence of yellow granules in the cell membrane or cytoplasm was considered positive TM4SF1 protein staining. Five locations in ovarian tissues without necrosis were randomly selected, and 100 cells in each field were observed under a microscope at 400X magnification. The score of each field was comprehensively determined according to the staining intensity and the number of positive cells. The scores were recorded and averaged to obtain the immunostaining score of each section. The standards of the staining intensity score were as follows: no color (−) was 0 point, light yellow color (+) was 1 point, yellow-brown color (++) was 2 points, and brown color (+++) was 3 points. The standards of the score of the number of positive cells were as follows: ≤5% was 0 points, 6%~ 25% was 1 point, 26%~ 50% was 2 points, 51%~ 75% was 3 points, and > 75% was 4 points. The product of these two scores > 3 was defined as positive TM4SF1 protein expression. All sections were independently reviewed by two experienced pathologists. The average value was obtained after double-blind scoring.

### The effect of TM4SF1 gene RNAi on the biological behaviors of HO8910PM and SKOV3 cells

#### Lentivirus-mediated transfection of HO8910PM and SKOV3 cells with shRNA

The lentiviral plasmid containing shRNA and the empty lentiviral plasmid were separately transfected into 293 T cells as an interfering virus particle package. The supernatant was collected and concentrated to obtain LV-TM4SF1-RNAi-Luc, LV-CON-RNAi-Luc. The virus concentrates were used to infect HO8910PM and SKOV3 cells at a multiplicity of infection (MOI) of 10. The enhanced infection solution (ENi.S) and 1640 culture medium were added. Cells with strong green fluorescence signals after 96 h of infection were sorted using a flow cytometer, cultured, and amplified. The amplified cells were LV-TM4SF1-RNAi-Luc/HO8910PM cells, LV-CON-RNAi-Luc/HO8910PM cells, LV-TM4SF1-RNAi-Luc/SKOV3 cells, LV-CON-RNAi-Luc/SKOV3 cells.

#### Detection of TM4SF1 mRNA expression in HO8910PM and SKOV3 cells using RT-qPCR after RNAi

The reaction parameters were as follows: 1 cycle of pre- denaturation at 95 °C for 30 s followed by 40 cycles of denaturation at 95 °C for 5 s and annealing and extension at 60 °C for 34 s. The data were analyzed using an Agilent MX-3000P instrument (Agilent Technologies, USA).

#### Detection of TM4SF1 protein expression in HO8910PM and SKOV3 cells using western blotting after RNAi

Cells were lysed in RIPA buffer to extract total cellular proteins. SDS-PAGE sample buffer was added, and the proteins were denatured at a high temperature and separated via electrophoresis. The proteins were transferred onto a PVDF membrane, and the membrane was blocked in 5% skim milk at room temperature for 1 h. The membrane was then incubated with the primary antibody (anti-TM4SF1, 1:2000; anti-β-actin, 1:1000) at 4 °C overnight and 1:5000 the secondary antibody (HRP-labeled goat anti-rabbit IgG, Beijing ZSGB-BIO, China) at room temperature for 1 h. Enhanced chemiluminescence (ECL) developing reagent was added, and the results were imaged using Gel Doc™ XR+ imaging system (Bio-Rad Laboratories, USA). The gray density value of the protein bands was analyzed using Image Lab 5.0 software. The experiment was repeated three times.

### The effect of RNAi targeting TM4SF1 gene expression on the growth and proliferation abilities of HO8910PM and SKOV3 cells

Cells at the logarithmic growth phase were treatment with pancreatic enzyme and inoculated onto 96-well plates at a density of 2 × 10^3^ (HO8910PM cells) or 6 × 10^3^ (HUVECs) cells/well. After cell attachment, MTT or CCK-8 reagent (DOJINDO, Japan) was added after 0 h, 24 h, 48 h, 72 h, and 96 h and incubated with cells at 37 °C for 1 h. The optical density (OD) values at 450 nm were detected using a microplate reader (Thermo, USA).

### Detection of the effect of RNAi targeting TM4SF1 gene expression on cell cycle in HO8910PM and SKOV3 cells using flow cytometry

Cells at the logarithmic growth phase were collected and fixed in 75% ice-cold ethanol at 4 °C overnight. According to the manual of the cell cycle detection reagent kit (Shanghai KeyGEN, China), cells were incubated with RNase A in a 37 °C water bath for 30 min, stained with PI at 4 °C in the dark for 30 min, and detected using a flow cytometer (EPICS XL, COULTER, USA).

### Detection of the effect of RNAi targeting TM4SF1 gene expression on colony formation of HO8910PM and SKOV3 cells using a colony-formation assay

After single cell suspension was prepared, cells were inoculated onto 6-well plates at densities of 100, 200, 400, and 600 cells/well. Each density was applied in 3 replicate wells. Cells were then incubated in a 37 °C and 5% CO_2_ incubator for continuous culture for 5–7 d. The cell culture was terminated according to the conditions of cell colony formation. Cells were fixed in methanol and stained with Giemsa stain. The cell colonies were counted under a microscope.

### Detection of the effect of RNAi targeting TM4SF1 gene expression on the migration ability of HO8910PM and SKOV3 cells using the migration test

Single cell suspension under starvation conditions was prepared using serum-free culture medium. Cells were inoculated into the top chamber of Transwell (8.0 μm, Costar, USA) at a density of 1 × 10^6^ cells. The bottom chamber of the Transwell was filled with 600 μl of culture medium containing 20% fetal bovine serum (FBS). Cells were cultured in a 5% CO_2_ incubator at 37 °C for 6 h, fixed in 4% paraformaldehyde (30 min at 25 °C), and stained with Giemsa staining solution for 30 min. Three random fields were photographed under an inverted microscope, and the cells that passed through the bottom chamber surface were counted. For each group, three replicate wells were prepared, and the experiment was repeated three times. The mean values were statistically analyzed ($\overline{x}$±SD).

### Detection of the effect of RNAi targeting TM4SF1 gene expression on the invasion ability of HO8910PM and SKOV3 cells using an invasion test

Single cell suspension under starvation conditions was prepared using serum-free culture medium. Cells were inoculated into the top chamber of Transwell coated with Matrigel (BD, USA) at a density of 1 × 10^6^ cells/well. The bottom chamber of the Transwell was filled with 600 μl of culture medium containing 20% FBS. Cells were cultured in a 5% CO_2_ incubator at 37 °C for 6 h, fixed in 4% paraformaldehyde (30 min at 25 °C), and stained with Giemsa staining solution for 30 min. Three random fields were photographed under an inverted microscope, and the cells that passed through the bottom chamber surface were counted. For each group, three replicate wells were prepared, and the experiment was repeated three times. The mean values were calculated ($\overline{x}$±SD).

### The effect RNAi targeting TM4SF1 gene expression on the formation of ovarian cancer cell-xenograft tumors in nude mice

Twelve nude mice were randomly divided into 2 groups with 6 animals in each group. Mice were labeled; group A was LV-CON-RNAi-Luc/HO8910PM, and group B was LV-TM4SF1-RNAi-Luc/HO8910PM. All animals were used in accordance with institutional guidelines, and the current experiments were approved by the Use Committee for Animal Care.

Cell suspension (100 μl) was subcutaneously inoculated into the right groin at a concentration of 1 × 10^8^ cells/ml. Tumor formation was observed every week, and the experiment was completed 6 w after the inoculation. Every week, the long (L) and short (S) diameters of the tumors were measured and the tumor volume was calculated according to the formula: V = L × S^2^/2.

Live imaging of xenograft tumors in nude mice was performed every 2 w for 6 w. The luciferase substrate Luciferin (Promega, Beijing, China) was intraperitoneally injected using a microinjector at 150 mg/kg. The growth of xenograft tumors in the mice were observed via In-Vivo Imaging System Fx Pro (BRUKER, USA). The luminescence value at each time point was quantitatively analyzed.

### Detection of TM4SF1 mRNA expression in xenograft tumors using RT-qPCR

Nude mice were euthanized with inhalation of carbon dioxide, and killing was completed by cervical dislocation. and the subcutaneous xenograft tumors were dissected and collected. TM4SF1 mRNA expression in xenograft tumors from the two groups was detected using RT-qPCR. The method was the same as that described in 2.2.2.

### Detection of TM4SF1 protein expression in xenograft tumors from each group using western blotting

TM4SF1 expression in xenograft tumors from the two groups was detected using western blotting. The method was the same as that described in 2.2.3.

### Statistical methods

All quantitative data were expressed as mean ± standard deviation ($\overline{x}$±SD). The Student’s t-test was used to compare quantitative variables. The Chi-squared test and Fisher’s exact test were used to compare categorical variables. Multivariate analysis was performed using COX proportional hazards regression model. SPSS v.16.0 software was used to statistical analysis. GraphPad Prism 5 Software was used to present graph. A value of *P* < 0.05 was considered statistically significant.

## Results

### Expression of TM4SF1 in different tissues and its association with clinical pathological characteristics and prognosis

#### The positive expression rates of TM4SF1 protein in ovarian tissues, epithelial ovarian tumor tissues, and matched lymph node metastatic foci

The positive expression rates of TM4SF1 protein in epithelial ovarian cancer tissues, ovarian benign tumor tissues, and normal ovarian epithelial tissues were 90.9, 65.2, and 31.3%, respectively, and all the differences were significant (*P* < 0.05). All (100%) metastatic lymph node foci and the corresponding primary foci were positive for TM4SF1 protein expression. TM4SF1 expression was observed in the cell membrane or the membrane of cells near the basement membrane in normal ovarian epithelial tissues and benign ovarian tumor tissues; however, the expression was mainly concentrated in the cytoplasm in cancer tissues (Fig. 1 and Table 4).

**Fig. 1:** TM4FS1 expression in ovarian tissues and metastatic lymph node foci detected by IHC (400X). **a** Positive control. **b** Negative expression of normal ovarian epithelial tissues. **c** Positive expression of normal ovarian epithelial tissues. **d** Positive expression of ovarian benign tumor tissues. **e** Positive expression of epithelial ovarian cancer tissues. **f** Positive expression of metastatic lymph node foci. Black arrows: Expression of TM4FS1 is concentrated in the membrane or near the basement membrane of the cell membrane; Red arrows: Expression of TM4FS1 is concentrated in the cytoplasm

**Table 4:** TM4FS1 expression in ovarian tissues and metastatic lymph node foci detected by IHC

Group	Total cases	Positive cases [positive ratio(%)]	χ^2^	*P* value
Normal ovarian epithelial tissues	16	5 (31.3)	–	0.022^*△^
Ovarian benign tumor tissues	23	15 (65.2)	5.969	0.015^**^
Epithelial ovarian cancer tissues	55	50 (90.9)	21.968	0.000^***^
Metastatic lymph node foci	30	30 (100)	–	–

* Normals VS Benigns; ** Benigns VS Cancers; *** Cancers VS Normals; △Statistic by Fisher’s exact probability test

#### The association between positive TM4SF1 protein expression and clinical pathological factors

Positive TM4SF1 protein expression (100%) was observed in epithelial ovarian cancer tissues from FIGO stage III-IV patients, which was higher than that in tissues from FIGO stage I-II patients (76.2%) (*P* = 0.012). The positive expression rate in ovarian cancer tissues with moderate to low differentiation was 97.4%, which was higher than that in those with high differentiation (75%) (*P* = 0.035). The positive expression rate of TM4SF1 protein was not significantly correlated with histological type or the amount of ascites (*P* > 0.05) (Table 5).

**Table 5:** TM4SF1 expression and Clinical pathology in ovarian cancer

Variates	Total cases	Positive cases [positive ratio(%)]	χ^2^	*P* value
FIGO			3.868	0.012
I~II	21	16 (76.2)		
III~IV	34	34 (100. 0)		
Histological grade			4.462	0.035
Grade 1	16	12 (75.0)		
Grade 2–3	39	38 (97.4)		
Histological type			–	0.398^△^
Serous	29	27 (93.1)		
Mucosity	16	15 (93.8)		
Endometrioid	8	6 (6/8)		
Clear cell	2	2 (2/2)		
Ascites			0.019	0.892
<500 ml	37	33 (89.2)		
≥ 500 ml	18	17 (94.4)		

△Statistic by Fisher’s exact probability test

#### The association between the positive expression rate of TM4SF1 protein in epithelial ovarian cancer tissues and clinical prognosis

Univariate and multivariate analysis results showed that the FIGO stage and histological grade were both influencing factors of ovarian cancer patient prognosis, and positive TM4SF1 protein expression was not an independent factor affecting the prognosis of ovarian cancer patients (P > 0.05) (Table 6).

**Table 6:** Univariate and multivariate analyses of factors influencing prognosis of ovarian cancer

Variates	Univariate analysis		Multivariate analysis	
	OR (95%CI)	P	OR (95%CI)	P
Age	0.81 (0.32–1.64)	0.368	–	–
FIGO	2.92 (1.53–6.06)	0.003	1.60 (0.97–9.40)	0.032
Histological grade	1.89 (0.93–3.57)	0.010	0.96 (0.61–6.34)	0.042
Ascites	1.07 (0.58–2.29)	0.046	1.02 (0.79–4.05)	1.193
TM4SF1	2.02 (1.00–7.89)	0.003	1.12 (0.68–9.46)	1.047

### The expression of TM4SF1 in HO8910PM and SKOV3 cells after RNAi

#### Screening of siRNA fragments that had the best silencing effect using RT-qPCR

Different gene silencing efficiencies were detected using fluorescence quantitative PCR. The results showed that all 3 of the siRNA constructs had inhibitory effects (*P* < 0.05). The gene silencing rate of the no. 813 gene fragment was 61.5%; which was better than that of the no. 733 (37.6%) and the no. 497 (28.6%) fragments (Fig. 2a).

**Fig. 2:** Expression of TM4SF1 in HO8910PM and SKOV3 cells after RNAi. **a** Expression of TM4SF1 interfered by different siRNAs. **b**, **d** Expression of TM4SF1 gene and protein in HO8910 after RNAi. **c**, **e** Expression of TM4SF1 gene and protein in SKOV3 cells after RNAi. *: *p* < 0.05 (Fig. 2a: * compared with control)

#### TM4SF1 gene expression in HO8910PM and SKOV3 cells after RNAi

The results of fluorescence quantitative PCR showed that TM4F1 mRNA expression (2-△△Ct) in the LV-TM4SF1-RNAi-Luc/HO8910PM group was significantly lower than that in the LV-CON-RNAi-Luc/HO8910PM group and the HO8910PM blank group [(0.05 ± 0.02) vs (0.91 ± 0.13)/(1.04 ± 0.13), *P* < 0.05] (Fig. 2b), TM4SF1 mRNA expression (2-△△Ct) in the LV-TM4SF1-RNAi-Luc/SKOV3 group was significantly lower than that in the LV-CON-RNAi-Luc/SKOV3 group and the SKOV3 blank group[(0.37 ± 0.07) vs (0.87 ± 0.06)/(1.01 ± 0.16), *P* < 0.05] (Fig. 2c).

#### TM4SF1 protein expression in HO8910PM and SKOV3 cells after RNAi

Western blotting results showed that the relative expression level of TM4SF1 protein in the LV-TM4SF1-RNAi-Luc/HO8910PM group was significantly lower than that in the LV-CON-RNAi-Luc/HO8910PM group and the HO8910PM blank group [(0.11 ± 0.01) vs (0.58 ± 0.02)/(0.65 ± 0.03), P < 0.05] (Fig. 2d), the relative expression level of TM4SF1 protein in the LV-TM4SF1-RNAi-Luc/SKOV3 group was significantly lower than that in the LV-CON-RNAi-Luc/SKOV3 group and the SKOV3 blank group [(0.27 ± 0.03) vs (0.54 ± 0.03)/(0.56 ± 0.04) P < 0.05/](Fig. 2e).

### The effect of RNAi on the biological behaviors of HO8910PM and SKOV3 cells

#### The effect of RNAi on the growth of HO8910PM and SKOV3 cells

The cell growth curve showed that the cell doubling times of the LV-TM4SF1-RNAi-Luc/HO8910PM group compared with LV-CON-RNAi-Luc/ HO8910PM group and LV-TM4SF1-RNAi-Luc/SKOV3 group compared with LV-CON-RNAi-Luc/SKOV3 group were not significantly different. (Fig. 3).

**Fig. 3:** The effect of RNAi on the growth of HO8910PM and SKOV3 cells. **a** Knockdown of TM4SF1 did not affect HO8910PM cells growth. **b** Knockdown of TM4SF1 did not affect and SKOV3 growth

#### The effect of RNAi on the cell cycle of HO8910PM and SKOV3 cells

The flow cytometry results showed that the percentage of cells in G1 phase in the LV-TM4SF1-RNAi-Luc/HO8910PM group was 53.23 ± 3.12, the percentage of cells in S phase was 32.16 ± 3.01, and the percentage of cells in G2 phase was 14.61 ± 4.32; these values were not significantly different from those of the negative control group (LV-CON-RNAi-Luc/HO8910PM) (Fig. 4a, b) .

**Fig. 4:** The effect of RNAi on cell cycle of HO8910PM and SKOV3 cells. **a** Cell cycle of LV-CON-RNAi-Luc/HO8910PM cells. **b** Cell cycle of LV-TM4SF1-RNAi-Luc/HO8910PM. **c** Cell cycle of LV-CON-RNAi-Luc/SKOV3 cells. **d** Cell cycle of LV-TM4SF1-RNAi-Luc/SKOV3 cells

The flow cytometry results showed that the percentage of cells in G1 phase in the LV-TM4SF1-RNAi-Luc/SKOV3 group was 30.74 ± 1.82, the percentage of cells in S phase was 42.77 ± 0.66, and the percentage of cells in G2 phase was 26.49 ± 1.48; these values were not significantly different from those of the LV-CON-RNAi-Luc/ SKOV3 group (Fig. 4c, d).

#### The effect of RNAi on the colony formation ability of HO8910PM and SKOV3 cells

After single cell suspension was seeded at a density of 200 cells/well and cultured for 7 d, scattered colonies were observed. The numbers of colonies formed in the LV-TM4SF1-RNAi-Luc/HO8910PM group (133.7 ± 5.7) and the negative control group LV-CON-RNAi-Luc/HO8910PM (137.3 ± 6.0) were not statistically different (*P* = 0.487) (Fig. 5a). The numbers of colonies formed in the LV-TM4SF1-RNAi-Luc/ SKOV3 group (124.7 ± 12.7) and the negative control group LV-CON-RNAi-Luc/ SKOV3 (138.0 ± 12.1) were not statistically different (*P* = 0.262) (Fig. 5d).

**Fig. 5:** The effect of RNAi on the colony formation, migration, invasion abilities of HO8910PM and SKOV3 cells. **a** Knockdown of TM4SF1 did not affect HO8910PM cells colony formation. **b** Knockdown of TM4SF1 inhibited HO8910PM cells migration. **c** Knockdown of TM4SF1 inhibited HO8910PM cells invasion. **d** Knockdown of TM4SF1 did not affect SKOV3 cells colony formation. **e** Knockdown of TM4SF1 inhibited SKOV3 cells migration. **f** Knockdown of TM4SF1 inhibited SKOV3 cells invasion. *p < 0.05, **p < 0.001

### The effect of RNAi on the cell migration and invasion ability of HO8910PM and SKOV3 cells

#### The effect of RNAi on the migration ability of HO8910PM and SKOV3 cells

The number of cells that passed through the membrane in the LV-TM4SF1-RNAi-Luc/HO8910PM group was 37.7 ± 3.8, which was significantly fewer than that in the negative control group (107.3 ± 5.1; *P* < 0.05) (Fig. 5b). The results obtained in SKOV3 cells similar to HO8910PM cells (183.6 ± 62.94 vs. 347.0 ± 24.07) (Fig. 5e).

#### The effect of RNAi on the invasion ability of HO8910PM and SKOV3 cells

The number of cells that passed through the Matrigel, which simulated the basement membrane, was 32.3 ± 3.1, and this value was significantly lower than that in the negative control group (88.0 ± 2.6; *P* < 0.001) (Fig. 5c). The results obtained in SKOV3 cells similar to HO8910PM cells (129 ± 20.84 vs. 347.4 ± 30.33) (Fig. 5f).

#### The effect of TM4SF1 gene silencing on xenograft tumor formation in nude mice

At 5–10 d after inoculation of ovarian cancer cell suspension, subcutaneous hard nodules were palpable at the injection sites in the nude mice in the two groups. After 2 w, bioluminescence signals in tumor cells were detected using a live imaging system. At 6 w after inoculation, the luminescence signal was the strongest; in addition, the activity of the mice was significantly reduced, and the body weights were significantly reduced at 6 w. At 6 w, the xenograft tumor volume in group B was significantly less than that in the control group (group A) [(2118.3 ± 176.42) vs (3546.20 ± 378.61), *P* < 0.05] (Table 7, Fig. 6a, b, c).

**Table 7:** Subcutaneous transplanted tumor volume of each group

Group	Volume mm^3^(($\overline{\mathrm{X}}$±S))						
	1 W	2 W	3 W	4 W	5 W	6 W	P(6 W)
A	7.40 ± 2.95	27.98 ± 5.06	162.66 ± 14.44	717.05 ± 65.50	1306.80 ± 273.10	3546.20 ± 378.61	
B	7.85 ± 1.20	26.81 ± 1.60	113.21 ± 19.18	341.95 ± 34.19	890.89 ± 62.61	2118.3 ± 176.42	0.000^**1**^

**Fig. 6:** The growth of xenograft tumor inhibited by RNAi. **a**, **c** Volume of xenograft tumor. **b** luminescence signal of xenograft tumor detected by live imaging system. **d** Expression of TM4SF1 gene in xenograft tumor. **e** Expression of TM4SF1 protein in xenograft tumor

### Detection of TM4SF1 gene expression in xenograft tumors in each group using RT-qPCR

After RNAi, TM4SF1 mRNA expression (2-△△Ct) in xenograft tumors was significantly decreased compared to that in the control group [(0.08 ± 0.02) vs (1.00 ± 0.13), P < 0.05] (Fig. 6d).

### TM4SF1 protein expression in xenograft tumors in each group detected with western blotting

After RNAi, TM4SF1 protein expression (relative gray density value TM4SF1/GAPDH) in xenograft tumors was significantly decreased compared to that in the control group [(0.11 ± 0.05) vs (0.87 ± 0.05), P < 0.05] (Fig. 6e).

## Discussion

TM4SF1, also known as tumor-associated antigen L6 (TAAL6), is a distant relative of the TM4SF family. Because it lacks the CCG motif in the large extracellular loop and the entire sequence homology with other 33 TM4SF family members, it is classified into a novel superfamily containing TM4SF5, TM4SF4, TM4SF18, and TM4SF20 [12]. Because of its high expression in various epithelial tumor tissues and low expression in benign tumor tissues, it is considered a potential immunotherapy target [7–11].

### The role of TM4SF1 in tumor invasion and metastasis

At least 34 TM4SF family members have been discovered in the human body. They play important roles in embryonic development, cell migration, adhesion, metastasis, and fusion. Different TM4SF genes are located on different chromosomes and encode 20–30 kD transmembrane proteins. To date, many tumor metastasis- and invasion-related studies have focused on CD9, CD81, CD82/KAI1, CD151, and TM4SF1.

It has been shown that an increase in TM4SF1 expression can promote the migration ability of epidermal keratinocytes [13]. Increased TM4SF1 protein expression can also increase the invasion ability of lung cancer cells, and an anti-TM4SF1 monoclonal antibody can significantly reduce the invasion ability of lung cancer cells [14]. Down-regulation of TM4SF1 gene expression using RNA interference technology can reduce the migration of prostate cancer cells and the metastasis ability of cervical cancer cells [15]. A recent study showed that hsa-miR-141 can effectively interfere with TM4SF1 expression in prostate cancer to inhibit prostate cancer cell invasion and metastasis, which describes a new carcinogenesis mechanism of TM4SF1 and suggests the potential of targeting TM4SF1 in gene therapy [16].

Our group performed immunohistochemistry and showed that the positive expression rate of TM4SF1 protein in epithelial ovarian cancer tissues was higher than that in benign ovarian tumor tissues and normal ovarian tissues. Moreover, the positive expression rate in benign ovarian tumor tissues was higher than that in normal ovarian tissues. The level of TM4SF1 protein expression also increased with an increase in the FIGO stage of epithelial ovarian cancer and a reduction in the differentiation level, indicating that the expression of TM4SF1 increased with abnormal hyperplasia and malignant transformation of ovarian epithelial cells and suggesting that TM4SF1 might participate in the occurrence and development of ovarian cancer. In addition, the positive expression of TM4SF1 protein in tissues in all metastatic lymph node foci and the matched primary loci indicated that TM4SF1 protein might be closely associated with tumor invasion and metastasis. Inhibition of TM4SF1 expression significantly inhibited the migration and invasion ability of HO8910PM and SKOV3 cells.

Otsuka et al. [17] applied internal cDNA microarray technology to detect genetic changes in colon cancer cell lines (SW 480 and SW 620) and 58 cases of clinically stratified colorectal cancer tissues, and the results showed that TM4SF1 gene expression was closely associated with the progression of tumor stage and might be a potential marker of metastasis.

Gordon et al. [18] reported that TM4SF1 was a negative regulatory gene in apoptosis of malignant pleural mesothelioma cells and could promote tumor cell growth. The results in this study showed that inhibition of TM4SF1 expression did not have a significant influence on cell cycle or cell growth and proliferation ability.

Chang et al. [19] showed that TM4SF1 and aminopeptidase N (CD13) co-localized in cells and formed a complex on the surface of lung cancer cells to affect cell migration ability, which further mediated lung cancer cell invasion and migration.

This study showed that TM4SF1 was localized in the cell membrane or the membrane of cells near the basement membrane in normal ovarian epithelial tissues and benign ovarian tumor tissues. However, its expression was concentrated in the cytoplasm in cancer tissues. These results were consistent with the results of Allioli et al. [15], who showed that TM4SF1 protein expression was mainly concentrated in the cytoplasm in prostate cancer and in the apical membrane in benign tissues. This localization change of TM4SF1 protein in different tissues might be associated with cancer cell invasion and metastasis.

The relevant mechanisms underlying the involvement of TM4SF1 in cancer cell invasion and metastasis are still not clear. Huang et al. [5] showed that TM4SF1 mediated tumor metastasis through regulation of the migration-associated genes MMP-2, MMP-9, and VEGF. A recent study showed that TM4SF1 could interact with discoidin domain receptor 1 (DDR1) promoted by collagen I. In addition, TM4SF1 could recruit syntenin2 and PKCa and activate PKCa to induce the noncanonical DDR1 signaling pathway to regulate metastasis of dormant breast cancer cells to multiple distant tissues [20].

Some researchers have also performed studies on the association between TM4SF1 and clinical prognosis. Kao et al. [14] showed that high TM4SF1 protein expression was significantly associated with postoperative early recurrence and a short survival period in lung squamous cell carcinoma and that increased TM4SF1 protein expression shortened the survival period in a tumor-bearing animal model. The results in this study showed that TM4SF1 protein expression in epithelial ovarian cancer at the late stage was higher than that at the early stage. However, the results of multivariate analyses showed that the positive expression rate of TM4SF1 protein was not an independent prognostic factor for epithelial ovarian cancer patients.

At the cell level, we showed that the TM4SF1 expression level was not significantly associated with cell growth and proliferation. However, the nude mice tumor formation experiment showed that inhibition of TM4SF1 expression in HO8910PM cells significantly inhibited the growth of xenograft tumors. The possible reason is that RNAi does not completely inhibit TM4SF1 expression.

Furthermore, it has also been shown that TM4SF1 is a target gene of androgen receptor [15]. Immunization with the cytotoxic T lymphocyte (CTL) epitope of TM4SF1 in HLA-A2 transgenic mice induced CTL immune responses to effectively inhibit the growth of tumor cells that expressed TM4SF1 [21].

## Conclusions

Because TM4SF1 has selective expression features in tumors, can mediate tumor cell growth and invasion, as well as metastasis, and is closely associated with anti-tumor immune responses, TM4SF1 is a potential target for anti-invasion and metastasis in ovarian cancer.

## Abbreviations

DAB: 3,3′-diaminobenzidine
DAPI: 4′,6-diamidino-2-phenylindole
EOC: Epithelial ovarian cancer
FBS: Fetal bovine serum
FIGO: International Federation of Gynecology and Obstetrics
FITC: Fluorescein isothiocyanate
HRP: Horseradish Peroxidase
ICC: Immunocytochemistry
PVDF: Polyvinylidene fluoride
RNAi: RNA interference
RT-qPCR: Quantitative real time polymerase chain reaction
SDS-PAGE: Sodium dodecyl sulfate polyacrylamide gel electrophoresis
TM4SF1: Transmembrane 4 superfamily 1
